# Validation of Hydraulic Mechanism during Blowout Trauma of Human Orbit Depending on the Method of Load Application

**DOI:** 10.1155/2021/8879847

**Published:** 2021-03-04

**Authors:** Marcin A. Zmuda Trzebiatowski, Paweł Kłosowski, Andrzej Skorek, Krzysztof Żerdzicki, Paweł Lemski, Mateusz Koberda

**Affiliations:** ^1^Department of Structural Mechanics, Faculty of Civil and Environmental Engineering, Gdańsk University of Technology, Gdańsk 80-233, Poland; ^2^Department of Otolaryngology, Faculty of Medicine, Medical University of Gdańsk, Gdańsk 80-210, Poland; ^3^Department of Ophthalmology, Faculty of Medicine, Medical University of Gdańsk, Gdańsk 80-210, Poland

## Abstract

The more we know about mechanisms of the human orbital blowout type of trauma, the better we will be able to prevent them in the future. As long as the *buckling* mechanism's veracity is not in doubt, the *hydraulic* mechanism is not based on equally strong premises. To investigate the correctness of the hydraulic mechanism's theory, two different methods of implementation of the hydraulic load to the finite element method (FEM) model of the orbit were performed. The intraorbital hydraulic pressure was introduced as a face load applied directly to the orbit in the first variant, while in the second one the load was applied to the orbit indirectly as a set of nodal forces transferred from the external surface of the eyeball via the intraorbital tissues to the orbital walls within the contact problem. Such an approach is aimed at a better understanding of the pattern for the formation of blowout fractures during the indirect load applied to the orbital bones. The nonlinear dynamic analysis of both numerical models showed that the potential fracture was observed in the second variant only, embracing a relatively large area: both medial and lower wall of the orbit. Interestingly, the pressure generated by the intraorbital entities transferred the energy of the impact to the orbital sidewalls mainly; thus, the nature of the mechanism known as the *hydraulic* was far from the expected hydraulic pressure. According to the eyeball's deformation as well as the areas of the greatest Huber-Mises-Hencky (H-M-H) stress within the orbit, a new term of *strut mechanism* was proposed instead of the *hydraulic* mechanism as more realistic regarding the investigated phenomenon. The results of the current research may strongly influence the development of modern implantology as well as affect forensic medicine.

## 1. Introduction

The investigation of potential human orbital blowout fracture patterns is crucial for the correct understanding of the head injury mechanics. Since the late fifties of the 20th century, two accepted theories are describing blowout fractures known as buckling and hydraulic mechanisms [1]. The first theory describes the process of fracture formation within an orbit as a result of an impact concentrated solely at the orbital rim (direct load applied to the orbital walls), while the second theory refers to the analogical process due to the impact applied solely at the human eyeball (indirect load acting at the orbital walls). The force of the impact presses the eyeball inwards of the orbit, causing the believed intraorbital hydraulic pressure growth, which primarily results in both lower and medial orbital wall damage [2].

As long as any controversy has not aroused around the essence of the buckling mechanism during previous studies [3–6], still, some descriptions of a sufficiently precise model of the hydraulic mechanism involving the set of intraorbital entities into cooperation (MOBOSE) are available in the literature. Until the works of Al-Sukhun et al. [7], as well as Patel et al. [6], and Foletti et al. [8, 9], other attempts were taken to model the hydraulic mechanism, but the role of the intraorbital tissues was omitted there. Nagasao et al. built their models basing on the hydraulic pressure applied to the internal faces of the orbital walls [10, 11]. On the other hand, in the later work of Schaller et al., the hydraulic mechanism was modeled as a contact problem between an eyeball and a human skull; however, the simulation did not include the presence of other intraorbital soft tissues [12]. Al-Sukhun et al. were the first who presented the model of a blowout injury involving the intraorbital tissues into consideration during the hydraulic mechanism simulation; nevertheless, their FEM model was not built basing on the real skull geometry (CT scans) [13]. On the contrary to them, in the latest work of Patel et al. [6], the human head model with the detailed ocular anatomy was used to determine the energy thresholds of the impact required to procure the orbital wall fracture both for the buckling and hydraulic mechanisms. However, the model was described rather superficially, without details necessary to repeat those calculations. On the other hand, Foletti et al. also presented the model of the human skull including the idealized eyeball and intraorbital tissues [9]. Nevertheless, the work was concentrated on blunt injury cases only, and also neither pure buckling nor the pure hydraulic mechanism of orbital blowout trauma was analyzed there. Moreover, none of the previous models is taking the cyclic change of the intraocular pressure into consideration when analyzing the impact. It may have been implemented by introducing an additional inner hydrostatic stress state inside the eyeball varying in time [14] or by detailing the eyeball's model and going down deeper into the tissue. Considering a highly advanced model of the human eyeball, it would be possible to introduce the intraocular pressure by distinguishing the blood vessels based on detailed magnetic resonance imaging (MRI) scans along with the simulation of a blood flow [15, 16]. Another option is to develop a porohyperelastic model of the eyeball to investigate how changes in the permeabilities of the eyeball's tissues imply the orbital blowout mechanics [17], using, for instance, similar techniques as other authors [18–21].

Considering the above, the main aim of the current study is to take a step towards the investigation of the real character of the hydraulic mechanism during orbital blowout fracture. Only the confrontation of the two different methods of the impact transfer to the orbit will help to determine if there is a convergence between the results obtained from the intraorbital hydraulic pressure applied directly and evenly to the inner faces of the orbital walls (MOBE) and the advanced model (orbital bone, orbital globe, and intraorbital tissue elements—MOBOSE) loaded indirectly via intraorbital tissues. What is also important, the destructive pattern, as well as the potential fracture area, was determined for both models, if possible. Furthermore, the current work should be considered as the continuation of studies held by the authors [4, 5, 22, 23] that targeted also at enriching previous investigations presented by other authors by modeling an impact affecting orbital walls as a set of nodal forces applied at the eyeball's surface and transferred by the soft tissue to the bones regarding the contact problem, what is the first such attempt known to the authors. Worth noting, the load application using a set of forces generates more problems with achieving the convergence of the solution in the nonlinear dynamic analysis on the contrary to the rigid body impact. That effect is especially visible when considering bodies having significantly different Young's moduli during the contact problem, which emphasizes the difficulty of the current analysis. It is crucial for better understanding the real character of the hydraulic mechanism what may result in the improved prevention of such injuries in the future.

## 2. Materials and Methods

### 2.1. FEM Model Description

In order to investigate two different patterns of hydraulic pressure implementation to the human orbit, two individual FEM models basing on the geometry of a real human skull were assembled using the MSC Apex software. The first of them was the MOBE comprising thin shell elements representing the bony structure of the orbit with adjacent parts of the facial skeleton. The orbital part of the MOBE, which was the main area of the current research, was built using FEM elements of the averaged size of 2 mm, while for the remaining part of the skull relatively larger elements of irregular size were used. On the other hand, the second model (MOBOSE) was the enhanced variant of the MOBE regarding the contact problem between the thin shell bone elements and relatively soft and incompressible intraorbital solid structures representing intraorbital tissues (muscles, nerves, vessels, and connecting tissues). To model those structures, a mesh using analogous element size to the orbital part of the skull was used. Moreover, the MOBOSE was enriched by introducing the orbital septum closing the intraorbital volume from the front.

The analyzed human skull section covering the left orbital region was composed of 3616 triangular thin shell elements. According to the thickness detection basing on the CT scans of healthy and past nontraumatic patients, the model was divided into miscellaneous zones having individual thicknesses. It applies especially to the orbital region which was meticulously diversified that way. The human eyeball was modeled as a homogeneous incompressible body using 5828 tetrahedron solid elements, while the intraorbital fat combined with nerves, vines, and extraocular muscles was assembled analogously using 7749 tetrahedron solid elements. Finally, the orbital septum was modeled using 238 triangular thin shell elements, whose role was to hold the intraorbital bodies inside the orbit during loading as well as to stabilize the eyeball. After the geometries of the MOBE and the MOBOSE were finally assembled, both of them were exported to the MSC Marc/Mentat software to perform further numerical simulations. Worth noting, the MSC Marc/Mentat® software is using dedicated solutions to avoid locking problem for the incompressible and near incompressible response [24].

Linear elastic isotropic material parameters were applied to each section of the two described models, basing on the authors' previous work [5] as well as on the data gathered from the literature (see Table 1). According to the mentioned work, Youngs' modulus of orbital bones was identified by the authors (*E* = 1.3 GPa) after obtaining the consent of the Bioethical Committee of the Medical University of Gdańsk, while the research was conducted under the guidelines contained in the Helsinki Declaration [25].

Hinged boundary conditions were applied to all nodes from the outer rim of the investigated skull section of MOBE and MOBOSE where it should be connected with the remaining part of the skull. The distance of fixed nodes was large enough to guarantee no influence of them on the orbital region behavior. For the MOBOSE, the eyeball was additionally stabilized by the fixed displacements in *X* and *Z* global direction both at the anterior and the posterior pole nodes to avoid numerical instability problems. The orbital septum was connected to the nodes from the orbital walls at its outer rim, while nodes from its inner rim were linked to adjacent nodes of the eyeball using 51 nodal links forcing the same displacements. Finally, the touching type of the contact problem in the node to segment variant was established in the MOBOSE between three different contact bodies: (a) the analyzed part of the skull including the orbit and the orbital septum, (b) the intraorbital tissues, and (c) the eyeball.

In the first approach, the direct hydraulic pressure inside the orbit was established in the MOBE by applying the normal load of 3.823 MPa to orbital bones' surface of all 1835 thin shell elements forming the orbit (see Figure 1) giving the equivalent total force of 14400 N. That force value corresponded to the doubled value of the kinetic energy necessary to destroy the orbital bone via the blowout [12], and it was used to determine the moment of the orbital load fracture during the hydraulic mechanism.

In the second approach, the set of 41 equal nodal forces was used to verify if the hydraulic pressure effect will also occur when the indirect load was applied to the orbit within the more complex model (MOBOSE) regarding the contact problem (see Figure 2). Analogously to the MOBE, the same total load value and the impulse shape was used, while the load direction was parallel to the Frankfort horizontal plane covering the area of cornea approximately in that case. To improve the convergence of the solution during the nonlinear dynamic analysis, both the orbit and the intraorbital tissues were connected by establishing common nodes in the area of their contact. Such simplification may be justified by the fact that the intraorbital fat tissue is connected to the orbital bone by the periosteum being the outer layer of the bone.

To model the impulse of the impact, the time-load function was defined as having the shape of an isosceles triangle (see Figure 3), to imitate the airbag inflation during a car accident [26, 27]. The impulse was growing linearly starting from 0 at the initial loading phase, and when it reached its peak for time *t* = 25 ms, the unloading phase started and decreased coming to zero at time *t* = 50 ms. Finally, the analysis was meant to stop while reaching time *t* = 100 ms, what enabled the observation of vibrations in both models after unloading.

Finally, both FEM models were analyzed using the nonlinear dynamic algorithm proposed by Houbolt in the small strain and large displacement variant [28]. The computations included the constant integration step of Δ*t* = 1.0 · 10^−4^ s, as well as the parameters *α* = 1.5644 · 10^3^ and *β* = 1.7180 · 10^−5^ of the Rayleigh damping [29]. To determine the fracture appearance in the orbit, the mean yield criterion of the Huber-Mises-Hencky (H-M-H) stress of 150 MPa was considered as the ultimate stress according to Nagasao et al. [3]. The adopted criterion resulted from the linear-elastic isotropic material model. The authors met difficulty of further orbital bone property identification due to the complex shape and the fragility of orbital specimens which made it impossible to perform more sophisticated tests on the testing machine.

### 2.2. Computed Tomography (CT) Scan Survey

The authors made a review of the Medical University of Gdańsk Clinical Centre's database regarding patients suffering the orbital wall trauma and having complete medical records available. The survey covered the period of 2014–2020, starting from the introduction of the digital database in the center. Each patient with diagnosed orbital wall trauma was inspected individually, regarding his/her clinical interview as well as CT scan analysis. If only each verified clinical interview indicated a strike localized at the eyeball and/or an orbital and ophthalmological trauma was found concurrently in the data, such individual case was classified as a potential hydraulic mechanism result. Finally, the selected group was separated from all orbital wall trauma cases basing on the above criteria.

## 3. Results

### 3.1. FEM Analysis

The nonlinear dynamic analysis of the indirect type of load application to human orbit during blowout trauma using the two different types of models (MOBE and MOBOSE) provided several interesting observations.

The first of them resulted from the analysis of displacements in both models at the times corresponding to the moment of their greatest values that was *t* = 25.0 ms in the case of MOBE or soon after at time *t* = 25.4 ms in the MOBOSE due to the contact interactions, according to the applied load impulse shape. Extremal values of displacements in the MOBE were observed both in the medial and lower wall, while the two separate compact areas of displacements' concentration might be distinguished there: one located at the medial and the second at the lower walls of the orbit (see Figure 4). The maximal displacement was localized at the medial wall and did not exceed the value of 5.74 mm, while within the second distinct concentration area at the lower wall the displacements barely reached half of that value. On the other hand, analyzing the MOBOSE not only the extremal displacements values were greater than those observed in the MOBE, but also the location of the highest displacement occurrence within the orbit was shifted towards the middle part of the lower wall (see Figure 5). The highest values of displacement observed in the lower wall did not exceed 8.30 mm, while in the medial wall the value of 5.81 mm was reached, which was still higher than that observed in the MOBE. It is also worth noting, unlike the MOBE, that the extremal displacements inside the orbit did not form two separated areas of concentration, but they merged into one compact area instead, covering both the bottom and medial walls.

Analyzing the H-M-H stress in both models, the disproportion between the outcomes observed in the MOBOSE and the MOBE was significant. Interestingly, the applied ultimate stress threshold of 150 MPa did not exceed in the MOBE (see Figure 6). The highest value of the H-M-H stress of 130.9 MPa was observed within the medial wall, while in the lower wall the H-M-H stress values barely reached 75 MPa. Moreover, analogous to the displacement analysis in the MOBE, two separate areas of the H-M-H stress concentration were detected. The first one located in the middle of the lower wall on both sides of the infraorbital groove was visibly smaller than the second one located in the medial wall. In contrast to the MOBE, the potential crack of the orbital bone including both medial and lower walls was observed in the MOBOSE as one continuous area (see Figure 7). The mentioned zone, where the applied ultimate stress threshold exceeded, may be seen as significant as covering 553 mm^2^ of the orbit at time *t* = 25.4 ms corresponding to the applied load's peak. Nevertheless, it should be emphasized that the potential crack zone analysis was only an approximation, due to the linear elastic model of the bone.

What is more interesting, four separate potential orbital fracture initiation points in the MOBOSE were found (see Figure 8). Chronologically, the very first presumption that the orbital bone fractured was observed for node no. 116 within the medial wall at time *t* = 10.3 ms. In other words, the potential destruction of the orbital bone structure may be expected soon after reaching the external total load value of 5932.8 N, assuming that the stress limit was established at the level of 150 MPa. The subsequent independent initiation point of the potential fracture within the orbit was observed for the coordinates corresponding to node no. 242 localized in the lower orbital wall on the lateral side of the infraorbital groove at time *t* = 15.2 ms. Consequently, it may be concluded that, when the applied value of the external load exceeded 8755.2 N, the risk of the next separate point initiating the fracture appeared. What is also interesting, after further 1.1 ms and 1.2 ms, other analogous individual initiation points were found. Both of them were localized within the lower wall. Chronologically, the first of them (node no. 244) was situated between the infraorbital groove and the medial wall, while the second one (node no. 141) was located similarly to node no. 242 between the infraorbital groove and the lateral wall in the deeper parts of the orbit. All individual fracture initiation points within the orbit, the time steps of the anticipated damage occurrence, and corresponding total load values causing the failure were summarized (see Table 2).

No less interesting were the displacements and the deformation of the intraorbital soft tissues (see Figure 9) in which the role in MOBOSE was the reception and subsequently the transmission of the load to orbit using the contact interactions. According to the significant difference between Young's moduli applied to the bony parts of the orbit and soft tissues, the deformation observed for both intraorbital bodies was significant in relation to surrounding bony structures. According to the displacement map, the highest of them were located in the anterior part of the eyeball, including the cornea region. The mentioned area was located directly under the set of point forces representing the external load, whereas a completely different situation occurred at the opposite pole of the eyeball. The lowest values of the obtained displacement within the eyeball were located at its posterior. Worth noting, the relatively smaller displacements were observed for the rest of the intraorbital tissues, especially for those located in the deeper parts of the orbital cone. On the other hand, analyzing the deformation of those two relatively soft intraorbital contact bodies, both of them proved the dominant role of the transverse direction of the displacement according to the applied load. Moreover, the posterior part of the eyeball tended to deform symmetrically as its anterior, towards the center of the globe. The deformation of the posterior part of the rest of the intraorbital tissues was visibly lower, and it may be seen as closely related to the deformation of the surrounding orbital walls, whereas the effect of the sphere's pressure on the deeper parts of the orbit was not observed.

### 3.2. CT Scan Analysis

Finally, in order to validate the current numerical results, the CT scan analysis was performed for all patients classified as suffering orbital wall trauma via the hydraulic mechanism. Basing on the data available at the Medical University of Gdańsk Clinical Centre, the investigated group included 15 males aged between 18 and 61, where the median was 37.5. All patients suffered simultaneous lower and medial wall fractures with and without dislocation of the fractured bone fragment into the maxillary and ethmoidal sinuses (see Figure 10). Eleven of them were victims of a fight, while the rest were injured by other accidents. Due to conducting the validation process for the FEM analysis, the numerical simulations of expected fracture areas were compared with real clinical cases, according to CT scans gathered in the study. The location of the real fractures coincided with the simulated ones, while the areas of potential fracture within the orbit were also similar depending on the force value applied to the model. Hence, the authors attempted to estimate the external load value and the corresponding energy of the impact needed to cause investigated real fractures. The detected fracture area for the patient (see Figure 10(a)) coincided with the simulated area corresponding to the dynamic load of around 9800 N applied to the MOBOSE (for time *t* = 1.70 ms of the performed FEM analysis), while for the second patient (Figure 10(b)) the anticipated dynamic load was around 11500 N (for time *t* = 2.00 ms). According to the above increments during the transient analysis, the total strain energies were calculated: 43.2 J and 60.0 J.

## 4. Discussion

The nonlinear dynamic analysis of the orbital region impact showed two different methods of load application: the first tested in the MOBE and the second tested in the MOBOSE. Naturally, the general concentration zones for the displacements and the extremal H-M-H stresses may be seen quite similar in both cases: the most interesting response occurs within the medial and lower walls only. Nonetheless, what differentiates those two models is the exact localization of both the highest displacements and the extremal H-M-H stresses. The highest displacement observed in the MOBE was within the medial wall exactly at the time corresponding to the load's peak, whereas the extremal displacement in the MOBOSE occurred in the lower wall on both sides of the infraorbital groove with the advantage of the medial wall side, soon after reaching the peak of the load due to the contact interactions. Not only the exact localization differs between those two models in the displacement context, but also the range of the obtained extremal values is considerable. The extremal displacement observed in the MOBOSE was about 45% higher than the analogous value observed in the MOBE, despite the same total load applied in both models.

Similar observations may be applicable during the H-M-H stress distribution comparison within both models. However, the general concentration zones, as well as exact localizations of the extremal values, are similar; a large disproportion was observed analyzing the obtained values for these two cases. The H-M-H stress did not exceed the accepted ultimate stress value (150 MPa) in the MOBE in contrast to the MOBOSE, where the potential fracture area, corresponding to the ultimate stress threshold, exceeds embraced significant parts of the lower and the medial orbital wall. Analyzing the MOBOSE, the H-M-H stress observed in the deeper parts of the orbital cone may be seen as negligible in comparison to values observed in the sidewalls of the orbit. The H-M-H stress concentrated mainly on the medial and lower walls, which were the thinnest parts of the human orbit.

Moreover, the potential orbital damage is expected to occur first of all on the medial wall for the hydraulic mechanism in MOBOSE at the time of 10.3 ms of the analysis that corresponds to the approximate total external load value of 5933 N. Another independent initiation point of the potential damage is expected to occur on the lower wall of the orbit after the next 4.9 ms of the analysis. Such a situation may take place no sooner than the external load reaches the value of 8755.2 N. Hence, a clear contrast may be perceived since no potential symptom of the damage was detected in the MOBE, even though the total load value of 14400 N was reached. At the time step, when the potential failure occurrence was observed in MOBOSE, the extremal H-M-H value in the MOBE has not exceeded the value of 54 MPa. The results obtained for both models do not match each other, which may be recognized as the first indication that during the impact applied at the eyeball simulating a potential accident, the hydraulic pressure inside the orbit may not be the correct reflection of the actual state.

The second and the most important circumstance explaining why the hydraulic pressure may not be present in the orbit during the application of the indirect load to the orbit (MOBOSE) is the character of the deformation of soft tissues, which is especially applicable to the human eyeball subjected to the external load directly. The incompressible body of the eyeball deforms in the transverse plane mainly, according to the direction of the external load which is affecting the eyeball sphere. Furthermore, the posterior part of the eyeball moved in the opposite direction than the load's current direction. The direct consequence of the observed effects is the pressure reduction in the posterior parts of the orbit. At the same time, the eyeball took the ellipsoid shape with the increase of stress close to the equator of the eyeball concerning the load direction.

Interestingly, the energies of the impact during the hydraulic mechanism causing the orbital wall damage reported by almost all other authors are unquestionably lower than those observed in the current work. Exempli gratia, according to simulations of Nagasao et al., the impact energy of 0.933 J is believed to initiate the fracture within the orbit for hydraulic mechanism [11], while the computations of Patel et al. showed that the impact energies causing both lower and medial wall fractures were from the range of 3.0–5.0 J [6]. On the contrary to the above values, the calculated total strain energy corresponding to the very first moment of exceeding the applied H-M-H limit in the current model (MOBOSE) was 16.4 J. Since any potential damage was not observed in the MOBE, the procedure of calculating the destructive impact energy was omitted for it. Worth noting, similar outcomes to the current observations were also reported by Foletti et al., who achieved the value of even 12.25 J as the kinetic energy required to initiate the blowout fractures within the orbit [9].

Moreover, a relatively high convergence was observed between the FEM results for the pure hydraulic mechanism (MOBOSE) and the analyzed real clinical cases for recorded areas of orbital bone fractures. Both FEM analysis and clinical cases reported lower and medial wall fractures occurring at once, while the area of documented fractures among investigated CTs varies for each case. This is due to the fact that each of those cases was individual, with a different force loaded at a different angle that could deviate from the Frankfort horizontal plane. Moreover, the mechanism of actual trauma might not have been a perfectly pure case where the entire energy of the impact was concentrated at the eyeball only.

## 5. Conclusions

Upon the observations resulting from the current analysis, the conception of Smith and Regan Jr. of two different theories describing patterns of orbital damage appearance during the blowout type of trauma, which are buckling and hydraulic mechanisms, may be considered as inaccurate [1]. As far as the buckling mechanism's name reflects the nature of such trauma adequately, the analogical statement cannot be justified in the hydraulic mechanism context. Due to the fact that the intraorbital pressure transfers the energy of the impact to the orbital sidewalls mainly, the mechanism commonly known as the hydraulic is far from the supposed hydraulic pressure definition, in fact. According to the eyeball's deformation as well as the areas of the greatest H-M-H stress within the orbit, a new term of *strut mechanism* was proposed by the authors instead of the commonly used name of the hydraulic mechanism as more realistic according to the investigated phenomenon.

Worth noting, the novel element of the current investigation is the successful attempt to model the blowout type of trauma as the orbit was loaded indirectly via the contact interactions of the intraorbital soft tissues subjected to the set of forces directly, unlike what other authors did such as Al-Sukhun et al. [7, 13, 30], Schaller et al. [12], Patel et al. [6], and Foletti et al. [8, 9]. Those models concern the blunt type of impact when a rigid/deformable body collided with a deformable model of a human skull. Such an approach adopted by those authors generated a fewer number of problems with achieving the convergence of the solution during the nonlinear dynamic analysis, which undoubtedly makes the current work the unique one in that sense.

The authors of this manuscript plan to carry out more in-depth analyses considering the use of solid models of the skull along with a more detailed mapping of the intraorbital soft tissues, including the variable intraocular pressure due to the blood flow to reflect the nature of the entire orbital system as accurately as possible. Moreover, the results of the current research may strongly influence the development of modern implantology as well as affect forensic medicine.

## Figures and Tables

**Figure 1:** MOBE under the face loads applied to shell elements inside the orbit.

**Figure 2:** MOBOSE model (contact bodies) under the set of nodal forces.

**Figure 3:** Load-time function of applied impulse.

**Figure 4:** Displacement map (mm) without the deformation within the analyzed thin shell skull part during time *t* = 25.0 ms (MOBE).

**Figure 5:** Displacement map (mm) without the deformation within the analyzed thin shell skull part during time *t* = 25.4 ms (MOBOSE).

**Figure 6:** H-M-H stress distribution (Pa) without the deformation within the analyzed thin shell skull part during time *t* = 25.0 ms (MOBE).

**Figure 7:** H-M-H stress distribution (Pa) without the deformation within the analyzed thin shell skull part during time *t* = 25.4 ms (MOBOSE).

**Figure 8:** Potential orbital fracture individual initiation points. H-M-H stress distribution (Pa) without the deformation within the analyzed thin shell skull part during time *t* = 18.5 ms (MOBOSE).

**Figure 9:** Displacement map (mm) for the sagittal cross section of the MOBOSE: (a) without deformation and (b) with deformation.

**Figure 10:** Exemplary CT scan analysis; red arrows indicate observed orbital wall fractures. (a) Male, 49, suffering both eyeball and orbital injury after boxing training with multifracture of the medial and lower walls of the left orbit. Bone fragment dislocated into maxillary and ethmoidal sinuses. (b) Male, 59, a fight victim suffering multifracture orbital trauma including both medial and lower walls of the right orbit with translocation of the bone fragment into maxillary and ethmoidal sinuses. Clinically diagnosed diplopia and damage of maxillary nerve (CN V_2_).

**Table 1:** Material properties applied to the FEM models of the human orbit's region.

Section of the model	Young's modulus *E* (N/m^2^)	Poisson ratio *ν* (-)	Density *ρ* (g/m^3^)
Orbital bone [5, 31, 32]	1.3·10^9^	0.33	1,610
Skull bone [3, 31, 33]	1.3·10^10^	0.33	1,800
Eyeball [31, 34]	5.0·10^5^	0.499999	1,000
Intraorbital tissues [31, 35]	1.0·10^4^	0.499999	9,70
Orbital septum [36–38]	5.0·10^5^	0.33	1,200

**Table 2:** Summary of the nonlinear transient analysis regarding the contact problem (MOBOSE).

	Initiation points of the potential orbital wall fracture			
	Lower wall (1) (node no. 141)	Lower wall (2) (node no. 242)	Lower wall (3) (node no. 244)	Medial wall (4) (node no 116)
Time of reaching the ultimate stress threshold (150 MPa) (ms)	16.4	15.2	16.3	10.3
Averaged load value corresponding to the potential fracture (N)	9500	8800	9400	5900
Impact energy required to cause the fracture (J)	41.0	35.4	40.6	16.4

## Data Availability

Data are available on request to the corresponding author.

## Additional Points

*Article Highlights*. (i) Verification of the *hydraulic* mechanism during the blowout fractures. (ii) Two different FEM models of the human orbital region investigated. (iii) Intraorbital soft tissues considered. (iv) Nonlinear dynamic FEM analysis regarding the contact problem. (v) Significantly different stress distribution in the orbit than the alleged hydraulic state. (vi) Introduction of a new term of *strut mechanism* of blowout fractures.
